The article "Hyperfractionation versus Conventional Fractionation of Preoperative Intensity-Modulated Radiotherapy with Oral Capecitabine in Locally Advanced Mid-Low Rectal Cancer: A Propensity Score Matching Study" was retracted in 2023. Reasons: signs of a paper mill; suspected computer-generated content; unreliable results or conclusions; concerns about the data.

# Hyperfractionation versus Conventional Fractionation of Preoperative Intensity-Modulated Radiotherapy with Oral Capecitabine in Locally Advanced Mid-Low Rectal Cancer: A Propensity Score Matching Study

**DOI:** 10.1155/2022/9119245

**Published:** 2022-04-11

**Authors:** Chen Shi, Yangzi Zhang, Yongheng Li, Jianhao Geng, Xianggao Zhu, Hongzhi Wang, Yong Cai, Weihu Wang

**Affiliations:** Key Laboratory of Carcinogenesis and Translational Research (Ministry of Education/Beijing), Department of Radiation Oncology, Peking University Cancer Hospital and Institute, Beijing 100142, China

## Abstract

**Purpose:**

In theory, the hyperfractionated radiotherapy can enhance biological effect dose against tumor and alleviate normal tissue toxicity. This study is to assess the efficacy and safety of preoperative hyperfractionated intensity-modulated radiotherapy (IMRT) with oral capecitabine in patients with locally advanced rectal cancer (LARC).

**Methods:**

We retrospectively screened patients with LARC from January 2015 to June 2016. Patients that received hyperfractionated IMRT or conventional fractionated IMRT were eligible in the hyperfractionation (HF) group or conventional fractionation (CF) group, respectively. The primary outcome was the complete response rate. Secondary outcomes included toxicity, postoperative complications, anus-reservation operation rate, local recurrence and distant metastases rate, overall survival (OS), cancer-specific survival (CSS), and disease-free survival (DFS).

**Results:**

335 patients were included in the analysis. The complete response rate for the hyperfractionated and conventional fractionated IMRT was 20.41% vs. 23.47% (*P* = 0.583). The anus-reservation operation rate was 68.37% vs. 65.31% (*P* = 0.649). There were no cases of grade 4 toxicity during radiotherapy; the rate of grade 3 toxicity and postoperative complications was both comparable between groups. However, in the CF group, more patients had a second operation due to complications (0.0% vs. 5.68%, *P* = 0.011). The cumulative local regional recurrence and distant metastases rates of the HF group and CF group were 5.10% vs. 9.18% (*P* = 0.267) and 22.45% vs. 24.49% (*P* = 0.736), respectively. The 5-year OS, CSS, and DFS in the HF group and CF group were 86.45% vs. 73.30% (*P* = 0.503), 87.34% vs. 75.23% (*P* = 0.634), and 70.80% vs. 68.11% (*P* = 0.891), respectively.

**Conclusions:**

The preoperative hyperfractionated IMRT with oral capecitabine, with an acceptable toxicity and favorable response and survival, could reduce the rate of secondary surgery.

## 1. Introduction

Rectal cancer, one of the most common malignant tumors, is usually occult in onset. Most rectal cancer patients have locally advanced or advanced-stage disease at the time of diagnosis. As the living standards improved in the recent years in China, so has the incidence of rectal cancer, while the age of onset has decreased [1]. As a result, exploring best modes of rectal cancer treatment has been considered a priority.

The article "Hyperfractionation versus Conventional Fractionation of Preoperative Intensity-Modulated Radiotherapy with Oral Capecitabine in Locally Advanced Mid-Low Rectal Cancer: A Propensity Score Matching Study" was retracted in 2023. Reasons: signs of a paper mill; suspected computer-generated content; unreliable results or conclusions; concerns about the data.

Preoperative concurrent radiochemotherapy followed by total mesorectal excision (TME) surgery has become the standard treatment for patients with locally advanced rectal cancer (LARC) [2–5]. As for the choice of synchronized chemotherapy regimen, studies have demonstrated that oral fluoropyrimidine, capecitabine, may be as effective as intravenous 5-FU in neoadjuvant treatment of LARC, with the added advantage of oral administration [6, 7].

Over the years, intensity-modulated radiotherapy (IMRT) is increasingly used to treat gross tumor with greater accuracy and lower risk of damage to normal tissue, compared to three-dimensional conformal radiotherapy (3DCRT) [8]. Since 2007, our center has adopted conventional fractionated concomitant boost IMRT (2.3 Gy/f for primary tumor and 1.9 Gy/f for pelvic lymphatic drainage areas, 50.6 Gy and 41.8 Gy in 22 fractions, a single fraction per day) combined with capecitabine for preoperative chemoradiotherapy in locally advanced, resectable mid-low primary rectal cancer patients [9]. To date, over 800 patients have been treated with this strategy, which is associated with favorable efficacy and tolerable toxicity.

From a radiobiological perspective, the hyperfractionated radiotherapy has such characteristics as shortened time of total dose be given and higher relative biological effectiveness. What is more, it does not increase normal tissue damage due to the lower dose of a single radiotherapy and the ability to give adequate repair time to normal tissue. Rectal cancer is a moderately sensitive tissue for radiotherapy, in which the hyperfractionated radiotherapy may provide comparable or improved local control with favorable tolerance.

Therefore, the combination of hyperfractionated radiotherapy and concomitant boost IMRT technology may further improve the pathological complete response (ypCR) rate and local control, while it does not increase the damage of normal tissue. Little research on the preoperative hyperfractionated IMRT in LARC patients has been published to date. This study was aimed at assessing the efficacy and safety of hyperfractionated IMRT, compared to conventional fractionated, with concomitant boost technique with capecitabine in LARC.

## 2. Materials and Methods

### 2.1. Patients

This is a historical cohort study, which retrospectively recruited patients with locally advanced, resectable mid-low primary adenocarcinoma of the rectum who had undergone preoperative IMRT from January 2015 to June 2016 in our center. This trial was approved by a relevant ethics committee, according to the Helsinki Declaration. All patients had given informed consent for chemoradiotherapy or for surgery before treatment.

The article "Hyperfractionation versus Conventional Fractionation of Preoperative Intensity-Modulated Radiotherapy with Oral Capecitabine in Locally Advanced Mid-Low Rectal Cancer: A Propensity Score Matching Study" was retracted in 2023. Reasons: signs of a paper mill; suspected computer-generated content; unreliable results or conclusions; concerns about the data.

Pretreatment evaluation included medical history, physical examination, complete laboratory tests, and preoperative staging. Complete laboratory tests included complete blood counts, urine and stool analysis, liver and kidney function tests, and gastrointestinal tumor markers. Preoperative staging included total colonoscopy, pelvic magnetic resonance imaging (MRI) scans or endoscopic ultrasound (EUS) combined with pelvic computed tomography (CT) scans, and chest and abdominal CT scans. In cases of staging discrepancy between the two modalities, the higher stage was recorded, following the guidelines from the seventh edition of the TNM staging standard of American Joint Committee on Cancer (AJCC).

### 2.2. Inclusion Criteria

All patients had histologically confirmed primary rectal adenocarcinoma, within 10 cm from the anal verge, with no evidence of distant metastases. The T/N classification was stage T3 or resectable T4 (R0 or R1 resection deemed possible) with any N, or any T with N1 or N2 disease. Patients presenting with T2N0 tumors located within 5 cm from the anal verge were also included. The age at diagnosis was between 18 and 80 years. Patients were required to have an Eastern Collaborative Oncology Group (ECOG) performance status of 0, 1, or 2, with adequate liver, kidney, and bone marrow function.

### 2.3. Exclusion Criteria

Patients with history of chemotherapy, surgery, pelvic radiation, or any other antitumor therapy were excluded. Patients with history of another malignancy within 5 years were also excluded. Other exclusion criteria included acute obstructive symptoms, unresectable disease with radical radiotherapy dose, or any serious comorbidities precluding chemoradiotherapy and surgery.

### 2.4. Treatment

All patients received preoperative concomitant boost IMRT combined with capecitabine. Patients underwent CT-based simulation with 5 mm slices in the supine position with a full bladder [10, 11]. An MRI scan was simultaneously performed to accurately define the extent of the tumor if without taboo. These scans extended from the upper edge of L4 vertebrae to below the perineum. Intravenous contrast was used. And a custom immobilization device was used to minimize setup variability. Daily patient positioning was performed using skin marks and weekly cone-beam CT (CBCT). The gross target volumes (GTV) and clinical target volumes (CTV) were contoured on the axial CT/MRI fusion scan slices. GTV was defined as primary rectal tumor and involved lymph nodes. The CTV was defined as primary tumor, mesorectal region, presacral region, mesorectal lymph nodes, lateral lymph nodes, internal iliac lymph node chain, and pelvic wall area [12]. The external iliac lymph nodes and inguinal lymph nodes were considered part of the CTV when these lymph nodes were involved. The superior border of pelvic fields was the L5–S1 interspace, and the inferior border was the bottom of the obturator foramen, or the anal verge for low-lying tumors [9]. The radiation dose was prescribed for planning gross target volumes (PGTV) and planning target volumes (PTV) by adding a 5 mm margin to the GTV and CTV, respectively. The boost to the primary tumor (GTV) was administered synchronously with the whole pelvis (CTV) radiotherapy. The 95% isodose line was planned to encompass the 95% PGTV and PTV as a planning objective. Five-field dynamic IMRT technique was used to shape the fields.

The article "Hyperfractionation versus Conventional Fractionation of Preoperative Intensity-Modulated Radiotherapy with Oral Capecitabine in Locally Advanced Mid-Low Rectal Cancer: A Propensity Score Matching Study" was retracted in 2023. Reasons: signs of a paper mill; suspected computer-generated content; unreliable results or conclusions; concerns about the data.

Patients eligible for hyperfractionation (HF) group received hyperfractionated IMRT with 2 dose levels simultaneously: 95% PGTV 51 Gy and 95% PTV 40.8 Gy in 34 fractions, 1.5 Gy and 1.2 Gy per fraction, 2 fractions with at least 8 hours interval per day. Treatment was delivered 5 times per week, over 23 days. In conventional fractionation (CF) group (control group), the patients received conventional fractionated IMRT with 2 dose levels simultaneously: 95% PGTV 50.6 Gy and 95% PTV 41.8 Gy in 22 fractions, 2.3 Gy and 1.9 Gy per fraction, a single fraction per day. Treatment was delivered 5 times per week, over 30 days.

The small bowel, bladder, and femoral heads were contoured and designated as organs at risk. Bladder constraints were V50 ≤ 35 Gy and V5 ≤ 50 Gy. Small bowel constraints were such that no more than 120 cm^3^ of the volume should receive more than 15 Gy, no more than 80 cm^3^ should receive more than 45 Gy, and no more than 20 cm^3^ should receive more than 50 Gy [13]. The constraints of femoral head were V50 ≤ 30 Gy and V5 ≤ 50 Gy^9^.

Capecitabine was administered at 825 mg/m^2^ orally twice daily, 5 days per week, during radiotherapy [7].

All patients underwent reassessment of clinical staging and resectability 6–8 weeks after completion of chemoradiotherapy. Patients with resectable tumors received TME surgery. As per the Habr-Gama and Memorial Sloan-Kettering Cancer Center (MSKCC) criteria, patients with clinical complete response (cCR) or near cCR could choose radical surgery, transanal local resection, or the “wait and see” strategy [14, 15]. The last category of patients was subject to regular follow-up, and remedial surgery was performed if local tumor regeneration occurred.

The article "Hyperfractionation versus Conventional Fractionation of Preoperative Intensity-Modulated Radiotherapy with Oral Capecitabine in Locally Advanced Mid-Low Rectal Cancer: A Propensity Score Matching Study" was retracted in 2023. Reasons: signs of a paper mill; suspected computer-generated content; unreliable results or conclusions; concerns about the data.

The choice between abdominoperineal resection and anterior resection was left to the discretion of the attending surgeon. Patients with low rectal cancer (defined as ≤5 cm from the anal verge) undergoing sphincter-preserving surgery also received prophylactic ileostomy.

Administration of adjuvant chemotherapy was individualized. The regimen of capecitabine or CapeOX for 4-6 months was both for recommendations [16–18].

### 2.5. Follow-Up

All patients were evaluated weekly for adverse events during chemoradiotherapy. Toxicities were analyzed according to the criteria for acute radiation injury of the Radiation Therapy Oncology Group (RTOG) and Common Terminology Criteria for Adverse Events (CTCAE), version 4.0.

Following antitumor treatments, patients were evaluated every 3 months for the first year, every 6 months for the second and third year, and annually for the fourth and fifth years. Posttreatment follow-up included measurement of complete blood counts, liver and kidney function tests, and gastrointestinal tumor markers, as well as total colonoscopy, chest X-ray or CT scans, abdominal ultrasound or CT scans, and pelvic CT or MRI scans.

### 2.6. Study Endpoints

The primary endpoint was tumor complete response rate, including ypCR and cCR rate. The secondary endpoints included toxicity, postoperative complications, R0 resection rate, sphincter-preserving surgery rate, downstaging rate, tumor response grading (TRG), local recurrence rate, distant metastasis rate, overall survival (OS), cancer-specific survival (CSS), and disease-free survival (DFS).

The TRG system was recommended by the National Comprehensive Cancer Network (NCCN) Guideline version 2.2019 Rectal Cancer modified from Ryan et al. [19–21]. The OS was defined as the time from the diagnosis of rectal cancer to the date of death from any cause or to last follow-up appointment. The CSS was defined as the time from diagnosis to rectal cancer-related death. The DFS time was defined as the time from diagnosis to the occurrence of local recurrence or any form of distant metastasis. Local regeneration after nonsurgical strategy or partial resection, which could undergo salvage radical resection, was not considered a regional recurrence and not counted as a positive event.

### 2.7. Statistical Analysis

Statistical analysis was performed with STATA version 13.0. Quantitative data were compared using independent sample *t*-tests or Wilcoxon rank-sum tests, based on the distribution of the variables. The chi-square test was used to compare the differences between the classification groups. We used the Kaplan–Meier method to estimate the OS, CSS, and DFS. The log-rank test was used to test for statistical significance. All statistical tests were two-tailed, and the *P* value < 0.05 was considered statistically significant.

The article "Hyperfractionation versus Conventional Fractionation of Preoperative Intensity-Modulated Radiotherapy with Oral Capecitabine in Locally Advanced Mid-Low Rectal Cancer: A Propensity Score Matching Study" was retracted in 2023. Reasons: signs of a paper mill; suspected computer-generated content; unreliable results or conclusions; concerns about the data.

### 2.8. Propensity Score Matching

The clinically important factors and variables associated with complete response rate as indicated in univariate Cox models (*P* < 0.10) were used for calculating propensity score matching (PSM). The covariates included were age, gender, BMI, comorbidities, history of smoking and drinking, ECOG scores, tumor gross and histopathologic types, the distance from the anal verge, clinical T and N stage, the status of mesorectal fascia (MRF), and extramural venous invasion (EMVI) (yes/no).

## 3. Results

In total, 335 patients were included. There were significantly more patients with ECOG 2 (0.76% vs. 1.96%, *P* = 0.001) and MRF involvement (12.31% vs. 25.98%, *P* = 0.003) in the control group. In the 196 matched pairs of patients generated by the PSM, all variables were well balanced between groups (Table 1, all *P* values > 0.05).

### 3.1. Toxicity during Chemoradiation

All patients received concurrent radiochemotherapy. The rate of radiotherapy and chemotherapy completion in the HF group and CF group was 98.47% vs. 98.52% (*P* > 0.999) and 96.95% vs. 97.06% (*P* > 0.999), respectively. All patients underwent toxicity evaluation. There were no cases of grade 4 toxicity in either group. Grade 3 toxicities included leukopenia [2 (1.53%) vs. 3 (1.47%), *P* = 0.988], neutropenia [2 (1.53%) vs. 2 (0.98%), *P* = 0.650], diarrhea [2 (1.53%) vs. 2 (0.98%), *P* = 0.650], and radiation proctitis [3 (2.29%) *vs.* 2 (0.98%), *P* = 0.383]. The rates of grade 1-2 toxicities were also comparable between the two groups (Table S1, all *P* values > 0.05).

### 3.2. Surgical Procedure and Complications

In the HF group, 113 patients underwent radical surgery and 4 patients with cCR selected “wait and see” strategy. In the CF group, 179 patients underwent surgery and 3 patients with cCR selected observation. Surgery was performed after a median interval of 67 days (41-127 days) and 64 days (37-148 days) in the HF group and CF group, respectively (*P* = 0.872). Among the patients who underwent surgery, 113 and 178 patients of the HF group and CF group had R0 resection (113/113 [100.00%] vs. 178/179 [99.44%], *P* = 0.788), respectively. The rates of sphincter preservation operation in the HF group and CF group were 64.60% and 60.89%, respectively (*P* = 0.524). Among the 181 patients with low rectal cancer (≤5 cm from anal verge) who underwent surgery, 90 patients received sphincter-preserving surgery with prophylactic ileostomy. The sphincter preservation operation rate for the low rectal in the HF group and CF group was 50.70% (36 out of 71) and 49.09% (54 out of 110), respectively (*P* = 0.832). In matched cohorts, there were also no statistical differences in the rate of radical surgery, R0 resection, and anus-reservation operation between the two groups (Table 2 (all *P* values > 0.05).

The article "Hyperfractionation versus Conventional Fractionation of Preoperative Intensity-Modulated Radiotherapy with Oral Capecitabine in Locally Advanced Mid-Low Rectal Cancer: A Propensity Score Matching Study" was retracted in 2023. Reasons: signs of a paper mill; suspected computer-generated content; unreliable results or conclusions; concerns about the data.

Among patients who received surgery, 28 (24.78%) and 44 (24.58%) patients of the HF group and CF group, respectively, developed postoperative complications (*P* = 0.970). However, the CF group had a higher rate of secondary surgery due to postoperative complications (0/113 [0.0%] vs. 8/179 [4.47%], *P* = 0.019). In matched cohorts, the control group still had a higher rate of secondary surgery (0/87 [0.0%] vs. 5/88 [5.68%], *P* = 0.011) (Table 2).

### 3.3. Tumor Response

Twenty-four and thirty-seven patients in the hyperfractionation and control group, respectively, acquired tumor complete remission (18.32% vs. 18.14%, odds ratio [OR] = 1.012, 95% confidence interval [CI] 0.574-1.787). In 196 patients selected through the PSM, the rates of tumor complete remission in the HF group and CF group were 20.41% vs. 23.47%, respectively (OR = 0.736, 95% CI 0.313-1.295).

According to the NCCN-TRG system, there were 20, 38, 52, 3 and 34, 60, 80, 5 patients with a score of 0, 1, 2, and 3, respectively, in the HF group and CF group, without significant difference. The primary tumor and lymph nodes downstaging rate of the HF group and CF group were 68.70% vs. 66.18% and 78.63% vs. 79.90%, respectively (*P* values > 0.05). In matched cohorts, there were also no differences in the T or N downstaging rates between the groups (Table 3).

### 3.4. Relapse and Survival

Up to November 2020, the median follow-up was 42.0 months in the hyperfractionation group (range 3.9–72.1 months) and 45.8 months in the control group (range 3.8–70.2 months) (*P* =0.322).

To date, cumulatively, there were 6 locoregional relapses and 28 systemic relapses in the hyperfractionation group and 22 locoregional relapses and 49 systemic relapses in the control group. Hyperfractionated RT showed a lower local recurrence rate (4.58% vs. 10.78%, *P* = 0.045). However, in matched cohort, hyperfractionated RT did not show this advantage of local control. Besides, there were no differences between the matched cohorts on distant metastasis rate. The 5-year DFS of the HF group and CF group was 70.27% vs. 68.99% (hazard ratio [HR] = 0.889, 95% CI 0.570-1.386) (Table 4).

During the follow-up, 14 and 29 patients, respectively, in the HF group and CF group, have died. The 5-year OS of the HF group and CF group was 78.40% vs. 81.32% (HR = 0.875, 95% CI 0.461-1.662). The 5-year CSS of the HF group and CF group was 79.93% vs. 82.94% (HR = 0.843, 95% CI 0.424-1.676) (Table 4).

The article "Hyperfractionation versus Conventional Fractionation of Preoperative Intensity-Modulated Radiotherapy with Oral Capecitabine in Locally Advanced Mid-Low Rectal Cancer: A Propensity Score Matching Study" was retracted in 2023. Reasons: signs of a paper mill; suspected computer-generated content; unreliable results or conclusions; concerns about the data.

In matched cohorts, the 5-year OS, CSS, and DFS between the two groups were 86.45% vs. 73.30% (HR = 0.763, 95% CI 0.594-2.885), 87.34% vs. 75.23% (HR = 0.815, 95% CI 0.529-2.845), and 70.80% vs. 68.11% (HR = 0.962, 95% CI 0.602-1.791), respectively (Table 4 and Figure 1). There were no statistically significant differences in the survival rates between groups.

## 4. Discussion

Preoperative concurrent radiochemotherapy based on capecitabine followed with TME surgery has become the standard treatment for patients with LARC [2–5]. However, the specific implementation of the radiotherapy process, covering the choice of radiotherapy technology and the segmentation mode of radiotherapy dose, is varied between different centers. With the update of radiotherapy technology, more and more centers use IMRT, which is characterized by increasing accuracy of higher-dose delivery in the tumor area while synchronously reducing the risk of damage to normal tissue, compared to 3DCRT with first pelvic field irradiation and then boosts to the tumor area.

Hyperfractionated radiotherapy, compared to the conventional fractionated radiotherapy, can give similar doses in a shorter period of treatment time and increase the relative biologically effective dose (BED) to gross tumor but may not increase normal tissue damage. There are few reports on preoperative hyperfractionated radiotherapy used for LARC. Movsas et al. illustrated the applicability of hyperfractionated radiotherapy in their single-arm studies [22–25]. In LARC, neoadjuvant hyperfractionated radiotherapy showed the favorable local control and OS. However, these studies were in the era of two-dimensional radiotherapy. In Marsh Rde et al.'s single-arm study, patients received preoperative 3DCRT with hyperfractionation and gained favorable short-term effects with tolerable acute toxicity [26, 27], whereas the sample size of the above two studies were relatively small (17 and 53 cases, respectively).

Another two studies compared preoperative hyperfractionated and conventional fractionated 3DCRT for LARC. In Ceelen et al.'s nonrandomized controlled study, hyperfractionated radiotherapy group showed lower pCR rate and sphincter preservation rate, which may be related to the absence of simultaneous chemotherapy and radiotherapy-surgical interval [28]. But the incidence of anastomotic leakage, pelvic recurrence rate, and 5-year OS was not statistically different between the hyper- and conventional fractionation groups. In another study, the only randomized controlled trial, RTOG-0012 study, showed that concurrent hyperfractionated (45.6 Gy in 38 fractions, 1.2 Gy per fraction, 2 fractions per day) and 5-FU chemoradiotherapy had a higher pCR rate than conventional fractionated (45.0 Gy in 25 fractions, 1.8 Gy per fraction, 1 fraction per day) chemoradiotherapy (30% vs. 26%) while lower 5-year OS and DFS (61% vs. 75% and 78% vs. 85%). But for T4 disease, the hyperfractionated group showed a higher 5-year DFS (87.5% vs. 71.4%). In addition to favorable short-term effect and survival, 3-4 grade nonhematologic radiochemotherapy acute toxicity in hyperfractionated group was relatively slight (38% vs. 45%) [29, 30].

The article "Hyperfractionation versus Conventional Fractionation of Preoperative Intensity-Modulated Radiotherapy with Oral Capecitabine in Locally Advanced Mid-Low Rectal Cancer: A Propensity Score Matching Study" was retracted in 2023. Reasons: signs of a paper mill; suspected computer-generated content; unreliable results or conclusions; concerns about the data.

In a word, hyperfractionation is feasible in neoadjuvant radiotherapy of LARC. However, little research on the hyperfractionated IMRT has been published to date. To the best of the authors' knowledge, the present study is the biggest comparison of hyperfractionated and conventional fractionated concomitant boost IMRT in LARC. In this study, except RT fractionation, other treatment regimens, including concurrent chemotherapy, radiotherapy-surgical interval, and operation principle, were concordant.

According to the computational formula of the BED (BED = *n*∗*d*∗[1 + *d*/*α*/*β* value] − *γ*/*α*∗[*T* − *Tk*], where *n* is as number of fractions, *d* is as dose of per fraction, *α*/*β* value of tumor is considered 10 and of normal tissues is considered 3, *γ*/*α* represents repair rate always considered 0.6 Gy per day, *T* represents total days of radiotherapy regimen, and *Tk* represents days of delayed proliferation always considered 7 days), the hyperfractionation RT slightly increased the BED value of primary tumor (49.1 Gy vs. 48.4 Gy) and significantly reduced the BED value of normal tissues in the target area (43.3 Gy vs. 50.1 Gy). As a result, the hyperfractionated IMRT described in this study may reduce normal tissue damage while ensuring treatment efficacy.

The results of this study, including rate of complete remission and 5-year DFS, were consistent with the results of RTOG-0012 study. What is more, our findings show better 5-year OS and fewer side effects of radiotherapy. In a word, in this study, the hyperfractionated and conventional fractionated preoperative concomitant boost IMRT both showed favorable safety and effectiveness in LARC. But there were no statistically significant differences between groups in this study of the tumor response rate, likelihood of complete remission, downstaging, R0 resection, or sphincter preservation. Among the 335 eligible patients, patients who received hyperfractionation IMRT showed lower cumulative local recurrence rate. Nevertheless, in the matched cohort, this result was not withstanding. These results about recurrence may be related to the more patients with MRF involvement in the control group before match. Anyhow, both RT fractionation regimens showed favorable tumor outcomes in this study, as evidenced by comparable survival rates.

The article "Hyperfractionation versus Conventional Fractionation of Preoperative Intensity-Modulated Radiotherapy with Oral Capecitabine in Locally Advanced Mid-Low Rectal Cancer: A Propensity Score Matching Study" was retracted in 2023. Reasons: signs of a paper mill; suspected computer-generated content; unreliable results or conclusions; concerns about the data.

Moreover, this study showed that in terms of acute radiotherapy toxicity, these two RT regimens were comparable. However, in patients who had postoperative complications, the conventional fractionation group had a higher rate of secondary surgery. The postoperative complications that need surgical treatment, such as anastomotic fistula or hemorrhage, rectovesical or rectovaginal fistula, or ileus, of which the events number in their CF group were always higher than that in the HF group (Table 2), tend to correlate with radiation target volume delivered to adjacent normal tissues. The lower risk of secondary surgery was consistent with the reduced BED of organs at risk in hyperfractionated group. Overall, hyperfractionation IMRT might be less likely to cause serious surgical complications in LARC than the conventional fractionation IMRT.

In addition, the hyperfractionated radiotherapy, which shortens the total number of treatment days (23 vs. 30 days), may have additional advantages in terms of public health economics. Among the daily admissions to our hospital, about 70% of patients are from other provinces, who always pay a lot for extra living expenses including room and board, hotel fees, and transportation costs. For these patients, shortened treatment days always means reduced living expenses. On the other hand, referring to the national charging standard, the cost of hyperfractionated radiotherapy (IMRT) does not increase too much because of the capped fee for 24-fractionated radiotherapy, even if the actual fractionations of radiotherapy are more than 24.

All in all, the evidence this paper presented may provide an appropriate option for the clinical practice of LARC in the field of radiation oncology. We believe that our study makes a significant contribution to the literature because little research on the combination of hyperfractionated radiotherapy and concomitant boost IMRT technology in LARC patients has been published to date.

Of course, this study has several limitations. Firstly, it was a retrospective study in which the information bias was inevitable. Secondly, we did not assess the long-term complications of radiotherapy or the differences in the quality of life of patient subject to different treatments. Next, the effect of adjuvant chemotherapy on recurrence, metastasis, and survival was also not assessed. Besides, according to literature data, extranodal extension (ENE) of nodal metastasis has emerged as an important prognostic factor in rectal cancer. However, whether the presence of ENE in patients with rectal cancer who receive preoperative chemoradiotherapy has impact on survival outcome is controversial [31, 32]. In this study, due to the lack of pathological findings of ENE in the lymph node metastasis after neoadjuvant chemoradiotherapy, we could not further determine whether ENE was an additional prognostic factor between the HF and CF group.

The article "Hyperfractionation versus Conventional Fractionation of Preoperative Intensity-Modulated Radiotherapy with Oral Capecitabine in Locally Advanced Mid-Low Rectal Cancer: A Propensity Score Matching Study" was retracted in 2023. Reasons: signs of a paper mill; suspected computer-generated content; unreliable results or conclusions; concerns about the data.

## 5. Conclusion

The hyperfractionated preoperative concomitant boost IMRT may be associated with favorable response and survival and reduced rate of secondary surgery due to postoperative complications compared to conventional therapy in LARC. It may be an appropriate option for these out-of-town patients who require cost savings.

## Figures and Tables

**Figure 1:** DFS, OS, and CSS curves in preoperative IMRT cohort. (a) DFS in overall population (*n* = 335); (b) DFS in matched cohorts (*n* = 196); (c) OS in overall population (*n* = 335); (d) OS in matched cohorts (*n* = 196); (e) CSS in overall population (*n* = 335); and (f) CSS in matched cohorts (*n* = 196). Abbreviations: DFS = disease-free survival; OS = overall survival; CSS = cancer-specific survival; IMRT = intensity-modulated radiotherapy; HF = hyperfractionation; CF = conventional fractionation.

**Table 1:** Baseline characteristics by preoperative IMRT cohort.

Variable	Overall population		*P*	Matched cohorts		*P*
	HF *n* = 131 (%)	CF *n* = 204 (%)		HF *n* = 98 (%)	CF *n* = 98 (%)	
*Age (years)*			0.219			0.702
≤40	9 (6.87)	6 (2.94)		7 (7.14)	5 (5.10)	
41-65	93 (70.99)	147 (72.06)		66 (67.35)	71 (72.45)	
≥65	29 (22.14)	51 (25.00)		25 (25.51)	22 (22.45)	
*Gender*			0.388			0.881
Male	87 (66.41)	126 (61.76)		63 (64.29)	64 (65.31)	
Female	44 (33.59)	78 (28.24)		35 (35.71)	34 (24.69)	
*BMI*			0.352^∗^			0.975^∗^
<18.5	4 (3.05)	5 (2.45)		3 (3.06)	4 (4.08)	
18.5-23.9	70 (53.44)	86 (42.16)		51 (52.04)	47 (47.96)	
24-26.9	33 (25.19)	63 (30.88)		27 (27.55)	28 (28.57)	
27-29.9	14 (10.69)	30 (14.71)		11 (11.22)	14 (14.29)	
≥30	3 (2.29)	10 (4.90)		3 (3.06)	3 (3.06)	
NA	7 (5.34)	10 (4.90)		3 (3.06)	2 (2.04)	
*Comorbidities*						
Hypertension	36 (27.48)	64 (31.37)	0.448	29 (29.59)	30 (30.61)	0.876
Diabetes	16 (12.21)	35 (17.16)	0.219	12 (12.24)	12 (12.24)	>0.999
CHD	8 (6.11)	9 (4.41)	0.490	3 (3.06)	6 (6.12)	0.497^∗^
Atrial fibrillation	5 (3.82)	4 (1.96)	0.321^∗^	1 (1.02)	2 (2.04)	>0.999^∗^
Cerebrovascular- disease	4 (3.05)	8 (3.92)	0.677	4 (4.08)	3 (3.06)	>0.999^∗^
Abdominal and pelvic surgery history	24 (18.32)	45 (22.06)	0.409	20 (20.41)	20 (20.41)	>0.999
Smoking history	62 (47.33)	92 (46.94)	0.945	44 (44.90)	48 (48.98)	0.567
Drinking history	42 (32.06)	63 (32.14)	0.988	29 (29.59)	40 (40.82)	0.100
*ECOG scores*			0.001			0.820^∗^
0-1	130 (99.24)	200 (98.04)		97 (98.98)	96 (97.96)	
2	1 (0.76)	4 (1.96)		1 (1.02)	2 (2.04)	
*Gross types*			0.140^∗^			0.828^∗^
Borrmann I	77 (58.78)	119 (58.33)		59 (60.20)	60 (61.22)	
Borrmann II	29 (22.14)	32 (15.69)		20 (20.41)	17 (17.35)	
Borrmann III	3 (2.29)	2 (0.98)		2 (2.04)	1 (1.02)	
Complex	22 (16.79)	51 (25.00)		17 (17.35)	20 (20.41)	
*Histopathologic types*			0.262^∗^			0.277^∗^
Well-differentiated	10 (7.63)	9 (4.41)		6 (6.12)	2 (2.04)	
Moderately differentiated	102 (77.86)	161 (78.92)		76 (77.55)	83 (84.69)	
Poorly differentiated	13 (9.92)	16 (7.84)		10 (10.20)	9 (9.18)	
Signet-ring cell	2 (1.53)	4 (1.96)		2 (2.04)	1 (1.02)	
Mucious adenocarcinoma	3 (2.29)	4 (1.96)		3 (3.06)	0 (0.00)	
Adenocarcinoma	1 (0.76)	10 (4.90)		1 (1.02)	3 (3.06)	
*Distance from anal verge*			0.553			0.165
≤5 cm	87 (66.41)	129 (63.24)		63 (64.29)	72 (74.37)	
5.1-10 cm	44 (33.59)	75 (36.76)		35 (35.71)	26 (26.63)	
*cT stage*			0.988^∗^			0.248^∗^
T2	4 (3.05)	6 (2.94)		2 (2.04)	2 (2.04)	
T3	99 (75.57)	151 (74.02)		72 (73.47)	83 (84.69)	
T4a	22 (16.79)	37 (18.14)		19 (19.39)	11 (11.22)	
T4b	6 (4.58)	10 (4.90)		5 (5.10)	2 (2.04)	
*cN stage*			0.198^∗^			>0.999^∗^
N0	6 (4.58)	4 (1.96)		4 (4.08)	3 (3.06)	
N1-2	125 (95.42)	200 (98.04)		94 (95.92)	95 (96.94)	
*MRF+*	16 (12.31)	53 (25.98)	0.003	15 (15.31)	12 (12.24)	0.534
*EMVI+*	10 (7.69)	8 (3.92)	0.137	8 (8.16)	5 (5.10)	0.389

Abbreviations: IMRT = intensity-modulated radiotherapy; HF = hyperfractionation; CF = conventional fractionation; BMI = body mass index; CHD = coronary heart disease; ECOG = Eastern Collaborative Oncology Group; c = clinical; MRF = mesoretal fascia; EMVI = extramural venous invasion. ^∗^Fisher's exact.

The article "Hyperfractionation versus Conventional Fractionation of Preoperative Intensity-Modulated Radiotherapy with Oral Capecitabine in Locally Advanced Mid-Low Rectal Cancer: A Propensity Score Matching Study" was retracted in 2023. Reasons: signs of a paper mill; suspected computer-generated content; unreliable results or conclusions; concerns about the data.

**Table 2:** Surgical procedure and complications in preoperative IMRT cohort.

Variable	Overall population		*P*	Matched cohorts		*P*
	HF *n* = 131 (%)	CF *n* = 204 (%)		HF *n* = 98 (%)	CF *n* = 98 (%)	
*Surgery*			0.692			0.817
Yes	113 (86.26)	179 (87.75)		87 (88.78)	88 (89.80)	
No	18 (13.74)	25 (12.25)		11 (11.22)	10 (10.20)	
*R0 resection*	113/113 (100.00)	178/179 (99.44)	0.788^∗^	87/87 (100.00)	87/88 (98.86)	0.635^∗^
*Anus-reservation operation*	73/113 (64.60)	109/179 (60.89)	0.524	67/87 (68.37)	64/88 (65.31)	0.649
*Complications*	28/113 (24.78)	44/179 (24.58)	0.970	21/87 (24.14)	23/88 (26.14)	0.761
Anastomotic fistula/hemorrhage	6/113 (5.31)	11/179 (6.15)	0.766	6/87 (6.90)	6/88 (6.82)	0.984
Rectovesical/rectovaginal fistula	0/113 (0.00)	4/179 (2.23)	0.161^∗^	0/87 (0.00)	3/88 (3.41)	0.246^∗^
Pelvic infection/abscess	5/113 (4.42)	11/179 (6.15)	0.529	5/87 (5.75)	7/88 (7.95)	0.563
Ileus	5/113 (4.42)	12/179 (6.70)	0.418	1/87 (1.15)	5/88 (5.68)	0.211^∗^
Perineal wound infection	8/113 (7.08)	14/179 (7.82)	0.815	8/87 (9.20)	7/88 (7.95)	0.769
Abdominal wound infection	1/113 (0.88)	6/179 (3.35)	0.255^∗^	1/87 (1.15)	4/88 (4.55)	0.368^∗^
Other infections^∗∗^	5/113 (4.42)	4/179 (2.23)	0.315^∗^	3/87 (3.45)	0/88 (0.00)	0.121∗
Other complications^∗∗∗^	4/113 (3.54)	4/179 (2.23)	0.715^∗^	1/87 (1.15)	0/88 (0.00)	0.497^∗^
*Complication treatments*			0.019^∗^			0.011^∗^
Conservative	28/28 (100.00)	36/44 (81.82)		21/21 (100.00)	18/23 (78.26)	
Operative	0/28 (0.00)	8/44 (18.18)		0/21 (0.00)	5/23 (21.74)	

Abbreviations: IMRT = Intensity-modulated radiotherapy; HF = hyperfractionation; CF = conventional fractionation. ^∗^Fisher's exact. ^∗∗^Other infections included urinary system infection and pulmonary infection. ^∗∗∗^Other complications included lower limb venous thrombosis, pulmonary thromboembolism, and acute myocardium infarction.

**Table 3:** Tumor responses in preoperative IMRT cohort.

Variable	Overall population		*P*	Matched cohorts		*P*
	HF *n* = 131 (%)	CF *n* = 204 (%)		HF *n* = 98 (%)	CF *n* = 98 (%)	
*cCR+ypCR*	24 (18.32)	37 (18.14)	0.966	20 (20.41)	23 (23.47)	0.583
*NCCN-TRG*						
TRG 0	20/113 (17.70)	34/179 (18.99)	0.795^∗^	18/87 (20.69)	21/88 (23.86)	0.417^∗^
TRG 1	38/113 (33.63)	60/179 (33.52)		26/87 (29.89)	25/88 (28.41)	
TRG 2	52/113 (46.02)	80/179 (44.69)		40/87 (45.98)	40/88 (45.45)	
TRG 3	3/113 (2.65)	5/179 (2.79)		3/87 (3.45)	2/88 (2.27)	
*Downstaging*						
Downstaging of primary tumor	90 (68.70)	135 (66.18)	0.631	64 (65.31)	63 (64.29)	0.881
Downstaging of lymph nodes	103 (78.63)	163 (79.90)	0.778	78 (79.59)	81 (82.65)	0.769

Abbreviations: IMRT = intensity-modulated radiotherapy; HF = hyperfractionation; CF = conventional fractionation; cCR = clinical complete response; pCR = pathological complete response; NCCN = National Comprehensive Cancer Network; TRG = tumor regression grading. ^∗^Fisher's exact.

**Table 4:** Tumor relapses and survivals in preoperative IMRT cohort.

Variable	Overall population		OR/HR	95% CI	*P*	Matched cohorts		OR/HR	95% CI	*P*
	HF *n* = 131	CF *n* = 204				HF *n* = 98	CF *n* = 98			
*Local recurrence*	6 (4.58)	22 (10.78)	0.397	0.157-0.997	0.045	5 (5.10)	9 (9.18)	0.532	0.172-1.648	0.267
*Distant metastasis*	28 (21.37)	49 (24.02)	0.860	0.508-1.456	0.574	22 (22.45)	24 (24.49)	0.893	0.578-2.170	0.736
*Cumulative relapses*	30 (22.90)	56 (27.45)	0.785	0.471-1.308	0.352	25 (25.51)	27 (27.55)	0.900	0.477-1.699	0.746
*Cumulative death*	14 (10.69)	29 (14.22)	0.722	0.366-1.424	0.346	12 (12.24)	13 (13.27)	0.912	0.473-1.845	0.830
*Survival*										
5-year DFS	70.27%	68.99%	0.889	0.570-1.386	0.604	70.80%	68.11%	0.962	0.602-1.791	0.891
5-year OS	78.40%	81.32%	0.875	0.461-1.662	0.684	86.45%	73.30%	0.763	0.594-2.885	0.503
5-year CSS	79.93%	82.94%	0.843	0.424-1.676	0.626	87.34%	75.23%	0.815	0.529-2.845	0.634

Abbreviations: IMRT = intensity-modulated radiotherapy; HF = hyperfractionation; CF = conventional fractionation; OR = odds ratio; HR = hazard ratio; DFS = disease-free survival; OS = overall survival; CSS = cancer-specific survival.

The article "Hyperfractionation versus Conventional Fractionation of Preoperative Intensity-Modulated Radiotherapy with Oral Capecitabine in Locally Advanced Mid-Low Rectal Cancer: A Propensity Score Matching Study" was retracted in 2023. Reasons: signs of a paper mill; suspected computer-generated content; unreliable results or conclusions; concerns about the data.

## Data Availability

The datasets used and/or analyzed during the current study are available from the corresponding author on reasonable request.

## Supplementary Materials

Supplementary Materials Table S1: toxicity during chemoradiation in preoperative IMRT cohort. Abbreviations: IMRT = intensity-modulated radiotherapy; HF = hyperfractionation; CF = conventional fractionation.
